# The Value of 320-Slice Spiral Computed Tomography Perfusion Imaging in Staging and Long-Term Dynamic Evaluation of Breast Cancer

**DOI:** 10.1155/2022/7442123

**Published:** 2022-07-21

**Authors:** Hequn Geng, Zhilin Zhang, Xiaochen Zhang, Zhandong Liang, Yong Li, Shujun Cui

**Affiliations:** ^1^Department of Medical Imaging, The First Affiliated Hospital of Hebei North University, Zhangjiakou, 075000 Hebei, China; ^2^Department of Radiotherapy, The First Affiliated Hospital of Hebei North University, Zhangjiakou, 075000 Hebei, China

## Abstract

The value of 320-slice spiral computed tomography (CT) perfusion imaging in staging and long-term dynamic evaluation of breast cancer was explored. 120 breast cancer patients who underwent preoperative CT examination and were confirmed by surgery and pathology were selected. All patients underwent preoperative TNM staging of breast cancer, with 120 cases in each stage. According to the results of 320-slice spiral CT, the postoperative pathology and surgical methods were compared and analyzed. CT diagnosis of breast cancer showed that T1 sensitivity was 71% and accuracy was 61%, T2 sensitivity was 74% and accuracy was 64%, T3 sensitivity was 94% and the accuracy was 84%, and the T4 sensitivity was 100% and the accuracy was 91%. The sensitivity of N1 stage was 71%, and the accuracy was 61%; and the sensitivity of N2 ~ N3 stage was 81%, and the accuracy was 76%. There were 7 cases of M1 with distant metastasis, the sensitivity was 71%, and the accuracy was 71%. At T1 stage, blood flow (BF) was 39.2 ± 16.7 mL/min/100 g, blood volume (BV) was 2.66 ± 1.4 mL/100 g, mean transit time (MTT) was 8.16 ± 2.7 s, and permeability surface (PS) was 16.6 ± 9.7 mL/min/100 g. 320-slice spiral CT perfusion imaging technology provided a new diagnostic mode for everyone, which can quantitatively identify breast cancer with multiple parameters, which was of great significance for clinical auxiliary diagnosis.

## 1. Introduction

Breast cancer is one of the most common malignant tumors in women worldwide, and accurate preoperative staging is the key to its treatment effect. Breast cancer accounts for about 20% of new cancers, and about 15% of the mortality rate [1]. Due to changes in people's lifestyles and reproductive patterns, its prevalence has continued to rise significantly in China in recent years, and it also tends to be younger [2]. Statistics show that the incidence of breast cancer in Beijing, China, is about 44/100,000, which is close to the incidence of moderately developed countries [3]. In addition, timely and accurate diagnosis of breast lesions, and given standardized treatment, can greatly reduce the mortality rate of patients, improve the survival rate of patients, and significantly improve the quality of life of patients [4]. Therefore, it is of great necessity and urgency to take early measures to prevent and closely monitor high-risk groups of breast cancer, and to achieve early detection, early diagnosis, and early treatment of breast cancer, and it will also bring great clinical and social value.

The role of imaging examinations in the screening and early diagnosis of breast diseases is crucial. The most common imaging examination methods include ultrasound, mammography, and magnetic resonance imaging (MRI) imaging techniques [5]. Ultrasound and mammography have certain defects in the detection and characterization of breast lesions. Although ultrasonography is inexpensive, easy to operate, and has high repeatability, it has limitations such as different resolutions of instruments, great differences in operator experience, and inconsistent objective diagnostic criteria [6]. Mammography is sensitive to radiotherapy and chemotherapy, but lesions located deep in the glands of dense breasts and multifocal lesions have poor display ability and are easy to be misdiagnosed and missed. Its sensitivity is about 68~91%, and its sensitivity to lesions in dense breast will be greatly reduced, about 48% [7]. Compared with MRI perfusion imaging, breast CT perfusion imaging has the advantages of being simpler and faster, and this technique can be used for quantitative examination in different body positions [8]. Because of its faster scanning speed than ordinary computed tomography (CT), helical CT can have multiphase scanning and reconstruction in any direction and can completely display the morphology and structure of lymph nodes, which significantly enhances the accuracy of preoperative staging of breast cancer [9]. Breast disease CT perfusion imaging technology can detect changes in breast morphology and hemodynamic changes at an early stage. According to the changes of various perfusion parameters, it can indicate the probability of the existence of early lesions, distinguish benign and malignant lesions, and further help determine the nature of lesions according to the differences in perfusion parameters between breast cancer and benign lesions (such as breast hyperplasia and fibroadenoma) [10–12]. The theoretical basis of CT perfusion imaging is the principle of radiotracer dilution in nuclear medicine and the central volume law (mean transit time (MTT) = blood volume (BV)/blood flow (BF)). It refers to the continuous multiple scans of the same slice at the selected slice while the contrast agent is injected intravenously, and the TDC of each pixel in the slice is obtained, which reflects the changes in the perfusion volume of tissues and organs [13].

Due to the increasing incidence of breast cancer patients, many complications, and poor prognosis, some patients are detected late, which brings serious life and economic burden to patients and the country. Therefore, it is necessary to take early measures to prevent and closely monitor high-risk groups of breast cancer, so as to achieve early detection, early diagnosis, and early treatment of breast cancer. This is important for improving patient outcomes and quality of life. It is very necessary and urgent to evaluate the value of 320-slice spiral CT perfusion scanning in the preoperative staging of breast cancer, the way and regularity of its metastasis, and its long-term dynamic evaluation. It will also bring greater clinical value and social value [14]. The objective of this work was to investigate the value of various perfusion parameters of breast cancer in the diagnosis of breast cancer by 320-slice spiral CT perfusion imaging, combined with the clinical data and pathological confirmation data of patients after surgery, so as to evaluate the value of 320-slice spiral CT perfusion in preoperative staging, metastasis pathway, regularity, and long-term dynamic evaluation of breast cancer, providing imaging basis for the diagnosis and treatment of breast cancer.

## 2. Materials and Methods

### 2.1. Research Subjects

Data of 120 breast cancer patients who underwent preoperative CT examination and were confirmed by surgery and pathology in hospital from January 2016 to January 2017 were included. Ages ranged from 25 to 58, with an average age of 42. The preoperative tumor node metastasis (TNM) staging of breast cancer was performed for all patients. There were 120 cases in each stage. Inclusion criteria were given as follows: patients with no allergy to iodine-containing contrast agents, patients with no renal insufficiency (creatine level < 1.5 mg/dL), patients with no pregnancy, and patients with complete image data. Exclusion criteria were set as follows: patients who were lactating and pregnant women and patients without pathological diagnosis. This work was approved by ethics committee of hospital, and the families of the patients included signed the informed consent.

### 2.2. Breast Cancer Pathological TNM Staging Criteria

The 7th edition of breast pTNM staging jointly developed by the American Joint Committee on Cancer (AJCC) and the Union for International Cancer Control (UICC) was adopted [15]. The criteria were as follows:

1. Primary tumor (T): Tx: primary tumor cannot be assessed; T0: no evidence of primary tumor; Tis: carcinoma in situ; T1: maximum tumor diameter ≤ 20 mm; T2: maximum tumor diameter > 20 mm and ≤50 mm; T3: maximum tumor diameter > 50 mm; and T4: direct invasion of the chest wall or skin regardless of tumor size
2. Regional lymph nodes (N): Nx: regional lymph nodes cannot be assessed; N0: no regional lymph node metastases on histological examination; N1: micrometastases; or 1-3 ipsilateral axillary lymph nodes; transfer; N2: 4-9 ipsilateral axillary lymph node metastasis; or clinically found ipsilateral internal mammary lymph node metastasis without axillary lymph node metastasis; N3: 10 or more ipsilateral axillary lymph node metastasis; or subclavian lymph node metastasis; or clinically found ipsilateral internal mammary lymph node metastasis, with 1 or more ipsilateral axillary lymph node metastasis; Or 3 or more ipsilateral axillary lymph node metastasis, with no clinical findings, ipsilateral internal mammary lymph node metastasis confirmed by sentinel lymph node biopsy; or ipsilateral supraclavicular lymph node metastasis
3. Distant metastasis (M): M0: no metastases were found on clinical and imaging examinations; M1: distant metastases detected by clinical or imaging methods, or metastases > 0.2 m confirmed by histology

### 2.3. Imaging Examinations

In this study, Toshiba Aquilion 320-slice spiral CT, double-barrel high-pressure syringe, and vitrea workstation were adopted. The patient was placed in the prone position, the chest-neck junction and abdomen were elevated, and both breasts sagged naturally. The scanning range was from the top of the armpit to the lower edge of the breasts. Initially, the plane was selected by plain scan, and the middle plane was selected at the center of the lesion. The scanning parameters were set as follows: 121 kV, 201 mA, delay 7 s, slice thickness 6 mm, and 90 consecutive scans per slice. In the same way (with the consent and supervision of the patient), the enlarged lymph nodes and metastases were selectively scanned, and the nonionic contrast medium was injected through the cubital vein with a flow rate of 4.0 mL/s and a total volume of 51 mL. The patient was breathing calmly throughout the perfusion scan. All patients underwent 320-slice spiral CT scan before surgery, and the pathology and scan results were compared after operation. TNM staging was determined by 2 senior radiologists based on preoperative CT findings.

### 2.4. Postprocessing of Images

Image postprocessing was performed using the body tumor perfusion software in the vitrea workstation. The thoracic aorta was defined as the input artery, and the lesion area was set as the region of interest to calculate the four perfusion parameters, including blood flow (BF), blood volume (BV), mean transit time (MTT), and permeability surface (PS), in the region of interest (ROI).

The segmentation of the tumor ROI was all performed by one professional physician, and two physicians were responsible for the interpretation of the clinical results of the patients. In this work, it only performed retrograde anatomy and deep feature extraction on the largest tumor lesion in each patient. The pulsed phase images were selected for segmentation analysis, because the enhanced breast adenoma lesions in the pulsed phase were significantly different from adjacent normal glandular tissues. To obtain the depth features, the ROI was manually delineated along the tumor boundary at the largest tumor slice on CT arterial-phase enhanced axial images.

### 2.5. Long-Term Evaluation

All patients underwent CT scan before the surgery, and the pathology and scan results were compared after the surgery. It should file and track all patients, instruct them to review regularly, perform perfusion scanning for breast cancer metastases, and summarize the final results of distant metastasis in 6 months, 1 year, and 1.5 years.

### 2.6. Collection of Clinical Data

Methods of checking blood routine indexes were described as follows. The routine blood tests of patients were performed using an automatic blood cell analyzer. The five blood routine indexes were collected, including white blood count (WBC), red blood count (RBC), platelet (PLT), neutrophil absolute value (NEU), and lymphocyte absolute value (LYM).

### 2.7. Statistical Analysis

All data were analyzed by SPSS 19.0 software. Numerical data were expressed as ($\bar{x}\pm s$), and categorical data were expressed as percentages. The data conforming to the normal distribution were analyzed by *t*-test and analysis of variance, and the nonnormally distributed data were analyzed by the Wilcoxon nonparametric test. The enumeration data were analyzed by the chi-square test. Correlation analysis was performed using the Spearman correlation analysis. *P* < 0.05 was considered statistically significant.

## 3. Results

### 3.1. Clinical Characteristics

120 patients were included in this work, ranging in age from 25 to 58 years, with an average age of 42 years. The differences in age, number of births, breastfeeding, and family history of breast cancer among breast cancer patients in T stage, N stage, and M stage were shown in Table 1. The differences between the blood routine indexes of breast cancer patients with different T stages and N stages were shown in Table 2.

### 3.2. Comparison of Perfusion Parameters in Different Stages of Breast Cancer Patients

The comparison of perfusion parameters (mean ± standard deviation) of breast cancer patients with different stages was shown in Table 3.

### 3.3. Examination Results

According to the new TNM staging criteria of the International Association against Cancer, the findings were as follows (Figure 1). In 41 cases of T1 stage, the lesions were enhanced on CT enhanced scan, and the lesions were small nodules or small round masses, less than 2.1 cm, the sensitivity was 71%, and the accuracy was 61%. 34 cases of T2 stage lesions were nodular or round-like, with diameters ranging from 2.1 to 5.1 cm, with blurred borders (some cases were still clear), and the length and thickness of the burrs varied. Enhanced lesions enhanced, CT value increased by 31~51 Hu, the sensitivity was 74%, and the accuracy was 64%. In 27 cases of T3 stage, the sensitivity was 94% and the accuracy was 84%. In 18 cases of T4 stage, the lesions invaded the muscle layer or chest wall, the sensitivity was 100%, and the accuracy was 91%. The CT value results of patients with different T stages were shown in Figure 2.

There were 63 cases in N0 stage (no lymph node metastasis) and 41 cases in N1 stage (ipsilateral axillary lymph node enlargement, and the sensitivity and accuracy were 71% and 61%, respectively. In 16 cases of N2 ~ N3 stage, the lymph nodes showed heterogeneous enhancement after CT enhanced scan, some showed ring enhancement, the CT value increased by 32-52 Hu (1 case had no enhancement). The sensitivity was 81%, and the accuracy was 76%. The above results were shown in Figure 3. The CT value results of patients with different N stages were shown in Figure 4.

There were 113 cases in M0 and 7 cases in M1. The supraclavicular lymph nodes of patients with distant metastases beyond the ipsilateral breast showed heterogeneous enhancement after enhancement, and the CT value increased by 31 to 51 Hu, with a sensitivity of 71% and an accuracy of 71%. Differences in CT values between patients with and without distant metastases were shown in Figure 5. The 6-month, 1-year, and 1.5-year follow-up results were as follows: 2 cases of distant metastasis at 6 months, 3 cases of distant metastasis at 1 year, and 3 cases of distant metastasis at 1.5 years, as showed in Figure 6. Among the 8 cases of metastases, 2 cases were transferred to the contralateral breast endolymphatic chain, the systemic lymph nodes were enlarged, 2 cases were bone metastases, 2 cases were brain-lung metastases, and 2 cases were bone-lung metastases.

## 4. Discussion

Most breast adenocarcinoma patients will undergo CT examination before surgery, which can not only be used to assess the extent of breast adenocarcinoma lesions. In addition, it can also detect the presence of metastases in many organs and bone masses such as distant skin, chest wall, regional lymph nodes (axillary, internal mammary, and supraclavicular lymph nodes), so as to make systematic preoperative clinical staging and arrange follow-up treatment plans [16]. 320-slice spiral CT is an auxiliary diagnostic imaging tool, which has strong clinical value in the preoperative evaluation of breast adenocarcinoma. Many studies have shown that multiscale and multifeature combination has strong predictive value than a single feature, and multifeature combination analysis is more conducive to individualized management of patients [17, 18].

The advantage of dynamic helical CT enhanced scanning lies in the use of multilayer structures at different scanning rates to reflect the layered structure [19]. 41 cases of early breast cancer in T1 stage in this work, obvious enhancement appeared in the arterial phase, and the CT value increased >4.1 Hu. The lesions in the parenchymal phase also enhanced significantly, and they regressed significantly in the equilibrium phase, but the lesions in T2 ~ T4 phases all enhanced in the equilibrium phase, so the arterial phase was used to detect early breast cancer. A study has shown that the CT value of advanced breast cancer is higher than that of early breast cancer [20]. In stage t4, the skin and chest wall are involved, the fat layer is blurred and disappears, and the ribs can be destroyed. The lymph nodes of each group in N staging were significantly enhanced in the arterial and venous phases after CT enhanced scanning, especially in the venous phase, and the CT value increased by 31~51 Hu [21]. 320-slice spiral CT perfusion is helpful for preoperative lymph node analysis.

A study dissected 1,248 axillary lymph nodes of 72 patients with breast cancer and found that axillary lymph nodes with a length of less than 5.1 mm still had a 10.1% metastasis rate, the LNM rate of 5.2-9.1 mm was 17.4%, and the LNM rate of 10.2-20.1 mm was 19.8%. In addition, the rate of LNM with a long diameter greater than 19 mm was 41%, and there was no correlation between lymph node metastasis and the size and histological grade of the primary tumor [22, 23]. Combining with the literature, it can be concluded that axillary lymph node diameter > 1.2 cm can be classified as metastasis, but lymph nodes < 1.2 cm cannot be excluded. Patients in M stage were supraclavicular LNM or distant metastasis in this work. 320-slice spiral CT has become a common method for diagnosing liver, lung, and supraclavicular lymph nodes in breast cancer patients. In this work, among the 8 cases of metastasis, 2 cases were metastasized to the contralateral breast endolymphatic chain, the systemic lymph nodes were enlarged, 2 cases were bone metastases, 2 cases were brain-lung metastases, and 2 cases were bone-lung metastases.

## 5. Conclusion

The results in this work showed that 320-slice spiral CT thin slice scan can be used for preoperative staging and long-term dynamic evaluation of breast cancer and can accurately assess the extent and location of breast cancer, as well as the condition of thoracic and axillary lymph nodes at one time. There were also many problems and deficiencies in this work. The sample size was relatively small, and more experimental people should be included, not in a single area or in a small area. Clinical trials should be conducted in multicenter, large-sample hospitals. In conclusion, 320-slice spiral CT can be used to assist in the diagnosis and evaluation of breast cancer and had reference value.

## Figures and Tables

**Figure 1:** Results of T stage under CT imaging.

**Figure 2:** CT value results of patients with different T stages.

**Figure 3:** Results of N stage under CT imaging.

**Figure 4:** CT value results of patients with different N stages.

**Figure 5:** CT values of patients with or without distant metastasis.

**Figure 6:** Results of distant metastasis on CT imaging.

**Table 1:** The general information of included patients.

Stage	Age (years old)	Number of births	Breastfeeding (cases)	Family history of breast cancer (cases)
T1	26-52	0-1 times	21	2
T2	27-58	1-2 times	19	1
T3	25-57	1-2 times	22	3
T4	24-55	0-1 times	18	2
N0	24-53	1-2 times	17	1
N1	26-54	0-1 times	20	2
N2-N3	25-52	1-2 times	18	2

**Table 2:** Differences in blood routine indexes of breast cancer patients with different T stages and N stages.

Stage	WBC (×10^9^/L)	RBC (×10^12^/L)	PLT (×10^9^/L)	NEU (×10^9^/L)	LYM (×10^9^/L)
T1	5.26	4.58 ± 0.3	226.5 ± 54.2	3.53	1.35
T2	5.47	4.66 ± 0.4	229.7 ± 50.3	3.92	1.54
T3	6.03	4.71 ± 0.3	231.8 ± 44.4	4.22	1.63
T4	6.67	4.78 ± 0.5	235.7 ± 56.7	4.51	1.87
N0	5.33	4.35 ± 0.7	227.5 ± 52.1	3.42	1.38
N1	5.46	4.58 ± 0.6	229.3 ± 45.7	3.87	1.79
N2-N3	6.82	4.62 ± 0.9	236.6 ± 38.2	4.46	1.88

**Table 3:** The comparison of perfusion parameters (mean ± standard deviation) of breast cancer patients with different stages.

Stage	BF (mL/min/100 g)	BV (mL/100 g)	MTT (s)	PS (mL/min/100 g)
T1	39.2 ± 16.7	2.66 ± 1.4	8.16 ± 2.7	16.6 ± 9.7
T2	40.5 ± 18.3	3.23 ± 1.6	8.88 ± 3.6	17.3 ± 8.9
T3	42.4 ± 16.9	3.85 ± 1.5	9.06 ± 3.8	18.7 ± 9.8
T4	45.7 ± 19.7	3.91 ± 1.4	9.43 ± 3.5	19.5 ± 9.5

## Data Availability

The data used to support the findings of this study are available from the corresponding author upon request.
